The article "Effects of lncRNA LINC01320 on Proliferation and Migration of Pancreatic Cancer Cells through Targeted Regulation of miR-324-3p" was published in 2021. Journal: J Healthc Eng.

# Effects of lncRNA LINC01320 on Proliferation and Migration of Pancreatic Cancer Cells through Targeted Regulation of miR-324-3p

**DOI:** 10.1155/2021/4125432

**Published:** 2021-12-23

**Authors:** Hua Meng, Kun Guo, Yun Zhang

**Affiliations:** Gastroenterology Department, Caoxian People's Hospital, Heze 274400, Shandong, China

## Abstract

**Objective:**

LINC01320 is a new oncogenic gene. Nevertheless, the effect of LINC01320 on pancreatic cancer (PC) is still unclear. This research aimed to seek the influence of LINC01320 on PC and its possible mechanism.

**Methods:**

RT-qPCR is used to test the LINC01320 in tissues and cells. Cell viability, apoptosis, migration, and invasiveness are detected to explore the role of LINC01320 in PC, and target genes are predicted by bioinformatics methods. The mechanism of action was further explored by transfection of specific siRNA, miRNA mimetics, or miRNA inhibitors. In order to verify the effect of LINC01320 in vivo, we carried out tumor xenotransplantation.

**Results:**

We conclude that LINC01320 is highly expressed in PC tissues and cell strains. LINC01320 high expression was bound up with a poor prognosis. LINC01320 gene knockout inhibited the growth, migration, and invasiveness of PC cells. In addition, LINC01320 is expressed by miR-324-3p, which is also supported by in vivo experiments.

**Conclusion:**

LINC01320 is highly expressed in PC, and it can suppress the growth and migration of PC cells through targeted regulation of miR-324-3p, which is expected to become a latent target for clinical treatment.

## 1. Introduction

PC, as the malignant tumor with the lowest survival rate in the digestive system, has the characteristics of invasive local infiltration and metastatic spread. Therefore, these characteristics result in an overall median survival time of <1 year and a 5-year survival rate of about 5% [1]. The data show that [2] the incidence rate is increasing every year and tends to be younger at the same time. Because of the strong concealment of PC in the early stage, patients often miss the early diagnosis [3]. The lack of specific and sensitive biomarkers limits the possibility of economic and effective screening for sporadic PC [4]. At present, most patients with advanced PC can only be treated with chemotherapy because they cannot undergo surgery. For the time being, although chemotherapy has improved the survival rate of patients, it still cannot achieve the ideal effect [5]. Therefore, it is of great clinical significance to illuminate the complex mechanism of pancreatic tumorigenesis and develop new strategies for early detection and therapy of PC.

We find a targeted binding locus between LINC01320 and miR-324-3p through online prediction. Previous research has found that miR-324-3p is poorly expressed in PC and is associated with PC patients' prognoses. LncRNA, as one of the members of noncoding RNA, is a kind of noncoding RNA with a length of more than 200 nucleotides [6]. Previous studies have found that [7] lncRNA cannot directly code proteins, and it is considered a waste product in the transcription process by scholars. However, in recent years, it has been reported that lncRNA can be used as a molecular signal to regulate transcription and act as a sponge for miR to induce the changes in the profile of downstream target genes [8]. Accumulated evidence has revealed that lncRNAs affect the pathogenesis of human diseases, including malignant tumors [9]. For example [10], LncRNA HOTTIP regulates the characteristics of cancer stem cells of human PC by regulating HOXA9. In addition, studies have also shown that [11] long noncoding RNA NORAD is a new competitive endogenous RNA, which can enhance epithelial-mesenchymal transition induced by hypoxia and facilitate the metastasis of PC. LINC01320 is a newly discovered lncRNA, and there has been no related research on LINC01320 before. However, we concluded that the LINC01320 in PC tissue increased through analysis of the GSE86436 chip, which suggested that LINC01320 might be a potential biological indicator of PC.

## 2. Methods and Materials

### 2.1. Database Analysis

We logged into the GEO database [12], downloaded GSE86436 (lncRNA) and GSE59856 (miR) chips, synthesized matrix files, analyzed the data using the Limma package, and extracted LINC01320. miR-324-3p and miR-496 expression data were used to draw pictures.

### 2.2. Collection of Samples

40 patients with ductal PC treated in our hospital from January 2016 to January 2018 were collected. During the operation, the patient's cancer tissues and adjacent tissues were obtained and sent to the laboratory for detection by liquid nitrogen transport. All patients in this test were diagnosed for the first time, and they had not received targeted antitumor therapy before. The expected survival time of the patients was more than 1 month, and all patients were not complicated with other tumors. This research was ratified by the Medical Ethics Committee of our hospital, and it was performed according to the Helsinki Declaration.

### 2.3. Cell Culture

PC cells (CFPAC-1, AsPC-1, L3.6pl, and Panc-1) and normal immortalized human pancreatic epithelial cell line (HPDE6C7) were all purchased from ATCC, USA. The repurchased cells were cultivated in DMEM (Sigma-Aldrich, St. Louis) and replenished with 10% fetal bovine serum (FBS; HyClone, Logan, the United States) and stored in a 5% CO_2_ moist incubator at 37°C.

### 2.4. Cell Transfection

miR-324-3p mimetic (miR-324-3p-mimics), inhibitor (miR-324-3p-inhibit), negative control (miR-mimics, miR-inhibit), LINC01320 small interfering RNA (siRNA) (si-LINC01320#1,2,3), and scrambling siRNA (si-NC) of LINC01320 came from RiboBio (Guangzhou, China). For cells transfection, cells were developed on 6-hole plates until 60% fusion was achieved, and then cells were transfected through miRNA, siRNA, or plasmid by Lipofectamine 2000 reagent (Invitrogen, Carlsbad).

### 2.5. qRT-PCR

Tissues and cells are collected, and total RNA is segregated from tissues and cells using TRIzol reagent (Invitrogen, Carlsbad, California, the United States). Next, cDNA was compounded using reverse transcription kits (Invitrogen, Carlsbad, CA, the United States) on the basis of the manufacturer's specifications. Amplification is conducted using SYBR Green PCR Kit and ABI 7500 PCR (Applied Biosystems). The reaction system and reaction conditions were configured on the basis of the manufacturer's specifications. U6 and GAPDH were applied as internal parameters. The sequence of qRT-PCR amplification primers is displayed in Table 1. 2^−△△Ct^ was used to calculate the change method of relative multiple [13]. All PCR assays were reduplicated 3 times.

### 2.6. WB Detection

Cells are broken through RIPA cell lysis buffer. BCA protein detection kit (Pierce, USA) is applied to quantitate the protein level of each cell lysate. The same amount of the protein sample is loaded onto 10% SDS-PAGE gel and then moved to the PVDF membrane. After sealing with skim milk, the membrane is cultivated with the first antibody was liquated in TBST buffer at 4°C overnight and then incubated with secondary antibody binding HRP at room temperature for 2-3 h. In the end, the images of protein bands are taken through a Tanon detection system using ECL reagent (Thermo).

### 2.7. CCK-8 Detection

The transfected cells are collected, resuspended, and adjusted to 1 × 10^4^ cells and then inoculated on 96-well plates. Cell proliferation ability is detected according to the manufacturer's manual by cell counting kit-8 (CCK-8) kit (Dojindo, Kumamoto, Japan). Optical density values are determined at 0, 24, 48, and 72 hours at a wavelength of 450 nm.

### 2.8. Transwell Experiment

The transfected cells are collected and placed in the superior cavity of transwell coated with Matrigel (8 *µ*m pore size; Corning Inc., USA), and DMEM added with 10% FBS is used as a chemotactic agent. Then, it is added to the lower chamber. After further culturing for 24 hours, the invasive cells on the film were dyed with 0.1% crystal violet for 30 minutes, and 5 fields were randomly selected under a microscope (LEICA) for quantification.

### 2.9. Flow Cytometry Detection

PC cells were adjusted to a density of 5 × 10^4^ cells/hole and inoculated into a 6-hole plate. The cells were transfected after adherence to the wall for 48 h. The cell culture was terminated after transfection for 48 hours. After PBS washing, cells were digested with 0.25% trypsinase and 0.02% ethylenediaminetetraacetic acid (EDTA), collected, and washed 3 times with PBS. 250 *µ*L of precooled PBS was put in each tube and mixed evenly, and then 750 *µ*L of precooled absolute ethanol was put and lightly fixed at −20°C overnight. Cells were centrifuged at 1000 rpm for 5 min to remove ethanol. The flow tube was inclined. PBS was added to cells along the wall and centrifuged 3 times. Cells were precooled at 4°C with 200 *μ*L of phosphate complex solution. Then, 200 *μ*L and 100 *μ*g/mL of propidium iodinate solution were added (prepared with phosphate and containing 25 *μ*g/mLRnaseA), mixed in darkness, and placed at room temperature for 30∼60 min. Flow cytometry was performed 2 hours later.

### 2.10. Double Fluorescein Report

Complementary DNA fragments containing wild-type (LINC01320-WT) or mutant LINC01320 (LINC01320-MUT) fragments were subcloned downstream of the luciferase gene in the psi-CHECK2 luciferase reporting vector. In the above steps, miR-324-3p simulation or miR-324-3p inhibitor was cotransfected (Invitrogen, USA) into HEK293 cells with LINC01320 reporter vector using transfection reagent. After transfection for 48 hours, the dual-luciferase reporting kit (Promega, USA) was applied to continuously test the activities of firefly and renin luciferase in cell lysates.

### 2.11. Coimmunoprecipitation (RIP)

Magna RIP RNA binding protein immunoprecipitation kit (MILLIALE, Billerica, MA) is employed for operation, and the operation steps were carried out according to the kit instructions. The specific steps are as follows: RB cells were broken in RIP lysis buffer. Then, cell lysate, RIP buffer comprising magnetic beads bound to human anti-Ago2 antibody, and normal mouse IgG (as negative control) were cultivated at 4°C for 4 hours to extract the coimmunoprecipitation RNA for qRT-PCR analysis.

### 2.12. Statistical Analysis

In this study, GraphPad 7 was used to draw the required pictures and data analysis. SPSS20.0 was used to analyze the independent prognostic factors of patients. Measurement data was represented by mean number ± standard deviation (means ± SD). The comparison between groups was conducted by an independent sample *t*-test. The counting data were represented by percentage (%). The chi-square test was expressed by *χ*^2^. One-way ANOVA was applied for comparison among multiple groups, expressed as F. LSD *t*-test was applied for pairwise comparison afterward. Repetitive measurement and analysis of variance were applied for expression at multiple time points, expressed as F. Bonferroni was used for posttest. Pearson test was used to analyze the correlation of each gene. K-M survival curve was used to draw the total survival condition of patients. A log-rank test was used for analysis. There was a statistical difference with *P* < 0.05.

## 3. Results

### 3.1. LINC01320 Was Highly Expressed in PC and Had Poor Prognosis

Firstly, in order to confirm the LINC01320 in PC, we analyzed the LINC01320 in GSE86436 chip. Through analysis, we found that LINC01320 expression increased in PC samples. Subsequently, qRT-PCR was used to detect tumor tissues of PC patients, and it was found that the LINC01320 in cancer tissues was higher than that in tumor-adjacent tissues. Patients were further separated into high and low expression groups on the basis of the median value of LINC01320 in cancer tissues of PC patients. Analysis of clinical and pathological data of LINC01320 and patients revealed that patients with LINC01320 high expression had low differentiation and high TNM stage (III + IV) and significantly increased the risk of lymphatic metastasis (Table 2). Survival analysis revealed that the overall survival rate of patients with LINC01320 high expression was obviously lower than that of patients with low expression. In addition, we detected the LINC01320 in PC cells by qRT-PCR. Compared with normal pancreatic cells, the LINC01320 in PC cells was significantly increased (Figure 1).

### 3.2. Downregulation of LINC01320 Could Suppress the Growth and Invasion of PC Cells and Facilitate Cell Apoptosis

In order to ascertain the effect of LINC01320 on the growth and metastasis of PC cells, we selected the cells with the most significant expression of LINC01320 for transfection (AsPC-1, PANC-1). Then, the growth of the cells was observed (Figures 2(a) and 2(b)). CCK-8 test showed that the growth activity of cells transfected with si-LINC01320#1 was significantly inhibited compared with si-NC (Figure 2(c)). Transwell test showed that the number of cell invasions transfected with si-LINC01320#1 was significantly reduced compared with si-NC (Figure 2(d)). This flow cytometry cell counting experiment found that transfection of si-LINC01320#1 induced apoptosis of cells (Figure 2(e)). This suggested that LINC01320 might be a latent target for the therapy of PC.

### 3.3. LINC01320 Acted as Sponge of miR-324-3p

In order to ascertain the miR that LINC01320 could combine, online prediction software starBase [14] and LncBase [15] were used for prediction. The results revealed the miR-324-3p and miR-496 (Figure 3(a)). To ascertain the miR-324-3p and miR-496 in PC, we analyzed the miR-324-3p and miR-496 in the GSE59856 chip. The results revealed that miR-324-3p was low expressed in the chip, but the miR-496 expression was not different (Figure 3(b)). qRT-PCR also revealed that miR-324-3p was reduced in PC patients, but the miR-496 expression was not different (Figure 3(c)). Through correlation analysis, it was found that miR-324-3p and LINC01320 were negatively correlated in PC tissues (Figure 3(d)), suggesting that there might be a target connection of LINC01320 with miR-324-3p. Therefore, we conducted a double luciferase report and RIP experiment. The results show that the fluorescence activity of LINC01320-WT could be inhibited by miR-324-3p-mimics (Figures 3(e)-3(f)), while both LINC01320 and miR-324-3p could be precipitated by Ago2 antibody (Figure 3(g)). In addition, we also found that the miR-324-3p in PC cells transfected with si-LINC01320#1 was inhibited (Figure 3(h)). These experiments demonstrated that LINC01320 could serve as a sponge for miR-324-3p.

### 3.4. Upregulation of miR-324-3p Could Suppress the Growth of PC Cells

At present, there has been no relevant research on the influence of miR-324-3p on the growth of PC cells. We transfected miR-324-3p-mimics into PC cells. Then, the CCK-8 experiment found that the growth activity of cells transfected with miR-324-3p-mimics was inhibited compared with miR-mimics, and the Transwell experiment found that cell membrane penetrations cases after transfecting miR-324-3p-mimics was significantly declined compared with miR-mimics. This flow cytometry counting experiment found that transfection of miR-324-3p-mimics induced apoptosis of PC cells, which revealed that miR-324-3p might be a therapy target for PC (Figure 4).

### 3.5. Downregulation of LINC01320 Could Offset the Promotion of miR-324-3p-Inhibit on the Growth and Metastasis of PC Cells

At the end of the research, we needed to determine whether LINC01320 could change the growth of PC cells by adjusting miR-324-3p. Therefore, we cotransfected si-LINC01320#1 and miR-324-3p-inhibit into PC cells. Then, the CCK-8 experiment showed that the proliferation activity of cells transfected with miR-324-3p-inhibit was obviously enhanced compared with miR-inhibit + si-NC, and the Transwell experiment found that cell membrane penetrations cases after transfecting miR-324-3p-inhibit was significantly increased compared with miR-inhibit + si-NC. This flow cytometry found that the apoptosis rate of cells transfected with miR-324-3p-inhibit was markedly lower than that of miR-inhibit + si-NC. We also found that the Bcl-2 protein was obviously increased, and the Bax and Cle-caspase-3 protein were significantly decreased after transfecting miR-324-3p-inhibit through WB detection, but the above results were reversed after cotransfecting into cells with si-LINC01320#1, which showed that LINC01320 could regulate the growth and metastasis of PC cells through targeted regulation of miR-324-3p (Figure 5).

## 4. Conclusion

This research was designed to explore the clinical value of LINC01320 in PC and provide latent targets for PC therapy. We have concluded that LINC01320 is highly expressed in PC patients, and it can inhibit the growth and metastasis of PC cells by adjusting miR-324-3p. It is expected to become a latent target for the therapy of PC.

## 5. Discussion

PC is the malignant tumor with the highest mortality rate. A recent tumor epidemiological survey [16] shows that the number of PC cases and deaths exceeded 400,000 in 2018. Therefore, we urgently need to explore potential targets for the therapy of PC. In this research, we confirmed, for the first time, that LINC01320 was highly expressed in PC, and the prognosis of patients with high expression was poor. In addition, we also found that LINC01320 could target miR-324-3p to improve the growth and metastasis of PC cells, and it was expected to become a latent target for the therapy of PC.

Previous studies have found that [17] lncRNAmiR competes for microRNA response elements (MREs), thus inhibiting miR synthesis from causing expression changes and further affecting its downstream target genes. Moreover, other studies have shown that [18–20] lncRNAs participate in cell proliferation, invasion, apoptosis, differentiation, and other processes, with certain regulatory effects. LINC01320 is located on human 2p22.3. In previous studies [21, 22], LINC01320 is only highly expressed in the lncRNA expression profile of endometrial carcinoma and the lncRNA expression profile of myocardial infarction. This study was the first to find that LINC01320 was highly expressed in PC, and it was also found that the overall survival rate of patients with high expression of LINC01320 was lower than that of the low expression group. This suggested that LINC01320 was expected to be a potential indicator of PC. To further ascertain whether LINC01320 affected the development of PC, we conducted cell experiments. After knocking down LINC01320, it was observed that the growth and invasion activity of cells were obviously suppressed compared with the control, and cell apoptosis was induced after knocking down LINC01320. This revealed that LINC01320 might become a potential target for the therapy of PC.

At present, much research has found that lcnRNA participates in the development of PC by regulating miR. For example, studies by Wei et al. [23] found that LncRNA XIST promotes the proliferation of PC through miR -133a/EGFR. In addition, studies by Gao [24] found that LncRNA ZEB2-AS1 facilitates the growth and invasion of PC cells by adjusting the miR-204/HMGB1 axis. For the purpose of exploring the mechanism of LINC01320, we predicted miR that downstream of LINC01320 could combine, and it was found that miR-324-3p and miR-496 might have targeted binding relationship with LINC01320 through starBase and LncBase prediction, respectively. At present, there are few studies on miR-324-3p and miR-496 in PC. Firstly, to ascertain the miR-324-3p and miR-496 in PC, the miR-324-3p and miR-496 were analyzed in GSE59856 and GSE53325 chips through the GEO database. The results uncovered that miR-324-3p was low expressed in PC samples, but miR-496 had no significant difference in PC samples. Therefore, we chose the miR-324-3p for the test. miR-324-3p is located on the human 17p13.1 chromosome. Previous research found that miR-324-3p is differentially expressed in gastric carcinoma [25], colon carcinoma [26], and breast carcinoma [27]. Previous research found that [28] miR-324-3p is bound up with the prognosis of PC. In this research, qRT-PCR revealed that miR-324-3p was low expressed in PC tissues and negatively correlated with LINC01320 in cancer tissues. In addition, the growth and invasion ability of PC cells were suppressed and the apoptosis rate increased after upregulation of miR-324-3p, which suggested that miR-324-3p was also a latent target for the therapy of PC.

At the end of the study, to ascertain the influence of LINC01320 regulating miR-324-3p on the growth and metastasis of PC cells, we conducted the cotransfection experiment. By observing the cotransfected cells, we found that the cell proliferation and invasion ability were enhanced, the apoptosis rate was reduced, the Bcl-2 protein was enhanced, and the Bax and Cle-caspase-3 protein were decreased after knocking down miR-324-3p. However, the results were reversed after cotransfection with si-LINC01320#1, which proved that LINC01320 could improve the growth and metastasis of PC cells by adjusting miR-324-3p. However, there are still some shortcomings in this research. First of all, we did not predict the target genes of miR downstream. Secondly, we only verified the relationship between LINC01320 and miR-324-3p through in vitro experiments. Whether LINC01320 has the same effect in vivo is unclear. Finally, for the diagnosis of PC by LINC01320, previous research strongly suggested that lncRNA has high clinical significance in PC diagnosis, while we did not explore the diagnostic value of LINC01320 in PC. Therefore, we hope to carry out more experiments and collect more samples in future research to improve our research results.

To sum up, LINC01320 is highly expressed in PC, and it can suppress the growth and migration of PC cells through targeted regulation of miR-324-3p, which is expected to become a potential target for clinical treatment.

## Figures and Tables

**Figure 1:** Relationship between expression and survival of LINC01320 in pancreatic cancer. (a) Expression of LINC01320 in pancreatic cancer from GSE86436 chip in GEO database. (b) qRT-PCR detection of relative expression of LINC01320 in tumor tissue of pancreatic cancer. (c) Relationship between LINC01320 and the overall survival rate of pancreatic cancer patients by K-M survival analysis. (d) qRT-PCR detection of relative expression of LINC01320 in pancreatic cancer cells. ^*∗*^*P* < 0.05,^*∗∗*^*P* < 0.01,^*∗∗∗*^*P* < 0.001.

**Figure 2:** Effect of LINC01320 on the growth of pancreatic cancer cells. (a) qRT-PCR was used to detect the relative expression level of LINC01320 after the construction of si-LINC01320. (b) qRT-PCR was used to detect the relative expression level of LINC01320 in cells transfected with si-LINC01320#1. (c) CCK-8 was used to detect the change of cell proliferation ability after transfecting si-LINC01320#1. (d) Transwell experiment was used to the change of cell invasion ability after transfecting si-LINC01320#1. (e) Flow cytometry was used to detect the change of cell apoptosis ability after transfecting si-LINC01320#1. ^*∗*^*P* < 0.05,^*∗∗*^*P* < 0.01.

**Figure 3:** LINC01320 targeting miR-324-3p. (a) starBase and LncBase jointly predicted the target gene of LINC01320. (b) Expression of miR-324-3p and miR-496 in GSE59856 chip. (c) qRT-PCR was used to detect the relative expression of miR-324-3p and miR-496 in pancreatic cancer tissues. (d) Pearson test was used to analyze the correlation between LINC01320 and miR-324-3p expression in tumor tissues of pancreatic cancer patients. (e) Targeted binding site of LINC01320 and miR-324-3p. (f) Double luciferase report confirmed that LINC01320 targeted miR-324-3p. (g) RIP experiment confirmed that both LINC01320 and miR-324-3p were precipitated by Ago2 protein. (h) qRT-PCR was used to detect the miR-324-3p relative expression in pancreatic cancer cells transfected with LINC01320#1. ^*∗*^*P* < 0.05,^*∗∗*^*P* < 0.01,^*∗∗∗*^*P* < 0.001.

**Figure 4:** Effect of miR-324-3p on growth of pancreatic cancer cells. (a) CCK-8 experiment was used to detect the change of proliferation ability of pancreatic cancer cells after transfecting miR-324-3p-mimics. (b) A Transwell experiment was used to detect the change of invasive ability of pancreatic cancer cells after transfecting miR-324-3p-mimics. (c) Flow cytometry was used to detect the apoptosis rate of pancreatic cancer cells transfected with miR-324-3p-mimics. ^*∗*^*P* < 0.05,^*∗∗*^*P* < 0.01.

**Figure 5:** Effect of LINC01320 regulating miR-324-3p-inhibit on the growth and metastasis of pancreatic cancer cells. (a) CCK-8 experiment was used to detect the change of proliferation ability of pancreatic cancer cells transfected with si-LINC01320#1 and miR-324-3p-inhibit. (b) Transwell experiment was used to detect the change of invasive ability of pancreatic cancer cells transfected with si-LINC01320#1 and miR-324-3p-inhibit. (c) Flow cytometry was used to detect the change of apoptosis rate of pancreatic cancer cells transfected with si-LINC01320#1 and miR-324-3p-inhibit. (d) WB was used to detect the apoptosis-related protein changes in cells transfected with si-LINC01320#1 and miR-324-3p-inhibit. ^*∗*^*P* < 0.05,^*∗∗*^*P* < 0.01.

**Table 1:** Primer sequences.

Gene	Upstream primer (5′-3′)	Downstream primers (5′-3′)
LINC01320	AGGGATCCTGCAGGTTGGTG	TGGCATGGTGCAGTAGGAACT
miR-324-3p	ACTGCCCCAGGTGCTGCTGG	GCGAGCACAGAATTAATACGAC
GAPDH	TCCAAAATCAAGTGGGGCGA	AGTAGAGGCAGGGATGATGT
U6	AACGCTTCACGAATTTGCGT	GTGACGTTTGGGTCAGGTGC

**Table 2:** Relationship between LINC01320 and pathological data of pancreatic cancer patients.

Factors		LINC01320 relative expression		*P*
		Low expression (*n* = 20)	High expression (*n* = 20)	
Age				0.206
	≥60 years old	12	8	
	<60 years old	8	12	

Gender				0.490
	Male	13	15	
	Female	7	5	

Tumor differentiation				0.025
	Well/middle differentiated	15	8	
	Poorly differentiated	5	12	

TNM stages				0.004
	I-II	15	6	
	III + IV	5	14	

Tumor size				0.525
	≥2 cm	12	10	
	<2 cm	8	10	

Nodal metastasis				0.011
	Metastasis	6	14	
	Nonmetastasis	14	6	

## Data Availability

The datasets used/analyzed during the current study are available from the corresponding author on reasonable request.
